# Effect of Kvass on Improving Functional Dyspepsia in Rats

**DOI:** 10.1155/2022/5169892

**Published:** 2022-06-28

**Authors:** Zhanmei Shao, Jidong Zhong, Yuming Fang, Yongqiang Ma

**Affiliations:** ^1^College of Forestry, Northeast Forestry University, Harbin, Heilongjiang Province, China; ^2^Qiulin Beverage Technology Co., Ltd., Harbin, Heilongjiang Province, China; ^3^Heilongjiang Key Laboratory of Grain Food and Grain Resources Comprehensive Processing, School of Food Engineering, Harbin University of Commerce, Harbin, Heilongjiang Province, China

## Abstract

Functional dyspepsia (FD) is a common digestive system disease, and probiotics in the treatment of FD have a good curative effect. Patients with gastrointestinal diseases often show a poor response to traditional drug treatments and suffer from adverse reactions. Kvass can be used as a functional drink without side effects to improve the symptoms of FD patients. The results showed that compared with those of the model group, the body weight and food intake of the treatment group were significantly increased (*P* < 0.05), and the gastric residual rate of the treatment group was significantly decreased (*P* < 0.05); the amount of pepsin in the treatment group was significantly higher than that in the model group (*P* < 0.05); a high dose of Kvass could increase the contents of ghrelin, motilin (MTL), and gastrin (GAS) in the plasma and decrease the contents of vasoactive intestinal peptide (VIP) in the plasma; the contents of ghrelin, MTL, and GAS in the gastric antrum were also increased in the high-dose group. Kvass beverage can significantly improve the gastrointestinal function of rats, which may be because it can improve the contents of ghrelin, MTL, GAS, and VIP in both the serum and gastric antrum by regulating the expression of short-chain fatty acids in the colon.

## 1. Introduction

Kvass is a popular low-alcohol (1% alcohol content) beverage in Russia, Ukraine, and other Eastern European countries. It is brewed by dry bread fermentation. Its color is similar to beer and is slightly red. At present, consumers are increasingly fond of natural drinks composed of traditional ingredients [1]. Kvass production adopts bioengineering technology, with Russian bread, hops, and maltose as the matrix, mixed with probiotics, lactic acid bacteria, and other bacteria. Kvass beverage contains amino acids, vitamins, lactic acid, and other nutrients, which can promote the health of the intestinal digestive system at all levels. Probiotics can inhibit the reproduction of harmful bacteria in the intestine [2, 3], reduce toxins [4], and promote intestinal peristalsis [5], so as to improve the intestinal function and defecation.

Gastrointestinal disorders include gastrointestinal motility disorders (GIMD) and functional gastrointestinal diseases (FGID) [6, 7], mainly involving gastroesophageal reflux disease (GERD), functional dyspepsia (FD), irritable bowel syndrome (IBS), and chronic constipation. At present, the incidence rate of gastrointestinal motility disorders is very high in China [8]. Due to the irregular and unhygienic diet, the proportion of people suffering from gastrointestinal disorders has reached 25.92% of the total population [9, 10]. The number of outpatients with gastrointestinal function disorders accounts for 40% of the total patients, which indicates serious human health effects [11]. In Japan [12], the prevalence rate of gastrointestinal motility disorders in the outpatients of hospitals is as high as 31% [13], and in the United States, the proportion of patients with digestive system diseases is as high as 40% [14]. Gastrointestinal motility disorders have become one of the key research subjects of public health worldwide.

FD is a group of symptoms including epigastric pain, epigastric burning, postprandial satiety, and early satiety. A large number of investigations show that in China, FD affects 5%–10% of the people. The gastrointestinal tract is composed of the lumen and sphincter; therefore, the pathogenesis of gastrointestinal disorders is often related to these two organs, such as gastrointestinal motility disorder and imbalance of gastrointestinal motility, and gastrointestinal kinin secreted by intestinal endocrine cells will cause FD. Motilin (MTL) is a kind of active peptide that can stimulate gastrointestinal smooth muscle [15]. It can promote the secretion of pepsin [16], improve gastric emptying rate, and shorten the time of food in the small intestine. Gastrin (GAS) is secreted by the G cells of the duodenal mucosa and gastric antrum and can regulate gastrointestinal peristalsis, promote gastric emptying, and stimulate gastric acid secretion [17]. Vasoactive intestinal peptide (VIP) is a brain intestinal peptide [18, 19] and is a neurotransmitter. It mediates the relaxation of the lower esophageal sphincter, promotes the synthesis of NO by target cells, and makes the smooth muscle diastolic. Liang et al. [20] made a FD rat model through starvation, tail suspension, anger, and forced swimming. When the model rats had gastrointestinal motility disorder, the levels of MTL and cholecystokinin (CCK) in the plasma were significantly lower than those in the control group. A study on a FD rat model induced by restraint stress found that Atractylodes essential oil can significantly promote gastric emptying and increase the plasma MTL level in FD rats [21]. Oikawa and others [22] have proved that Banxia Houpu Decoction (HKT) can improve abdominal swelling and reduce intestinal gas in FD patients.

At present, the main drugs used in the treatment of FD are proton pump inhibitors (PPI), other acid inhibitors [23], prokinetic agents, and neuromodulators for visceral hypersensitivity, probiotics, and herbal therapy [24]. However, there is no drug on the market to treat all patients with FD, and the drugs have side effects on FD patients. Although FD is not a life-threatening disease, many outpatient studies show that FD obviously damages the quality of work and life of patients and brings huge economic burden to the medical system [25]. In order to alleviate this problem, we should take measures to alleviate the symptoms of FD in our daily life.

Recently, researchers found that probiotics may be beneficial to the treatment of FD patients. After probiotics enter the intestine, they increase the abundance of intestinal microorganisms, and the intestinal microbiota can inhibit the synthesis of bile acids in the liver [26], so as to reduce the secretion of bile acids from the duodenum, so as to relieve upper abdominal symptoms. As a drink containing a variety of probiotics, kvass can effectively alleviate this symptom.

The purpose of this study is to explore the ability of kvass to alleviate the symptoms of FD and to explore the pharmacological effects of Kvass on gastrointestinal hormones and brain gut peptides in FD rats, particularly, the indexes related to FD, including body weight, food intake, plasma ghrelin, MTL, GAS, VIP, and other routine indexes. Meanwhile, the expression of short-chain fatty acids in the colon was detected. The mechanism of Kvass in relieving FD in rats was elucidated. It lays a really good foundation for the treatment of patients with functional dyspepsia in the future.

## 2. Materials and Methods

### 2.1. Materials and Chemicals

#### 2.1.1. Bread Fermented Beverage

The beverage produced by simultaneous fermentation of yeast and lactic acid bacteria (independent separation) is a commercial product (called Kvass) prepared by Harbin Qiulin Beverage Technology Co., Ltd., with high concentration dilution technology. In short, mix bread flour (add 0.6 L neutral protease and 0.5 L per ton *β*-glucanase) and water in the ratio of 1 : 2.8, add saccharifying solution (pH 5.4) to saccharify for 3 hours, add yeast and lactic acid bacteria (inoculation amount 6%) to ferment for 48 hours, sterilize at 120°CUHT for 5 s, and then have it canned (500 mL/bottle).

#### 2.1.2. Materials and Instruments

The ELISA kits for rat MTL, GAS, VIP, and ghrelin were purchased from Nanjing Jiancheng Technology Co., Ltd. (Nanjing, China). The other reagents were domestic and of analytical grade.

An ultrapure water meter (Millipore, USA), an Al104 electronic analytical balance (Shanghai METTLER TOLEDO Instrument Co., Ltd.), a Yp10002 Matou electronic balance (Shanghai Guangzheng Medical Instrument Co., Ltd.), a Tgl-5-a high-speed centrifuge (Shanghai Anting Analytical Instrument Co., Ltd.), a Varioskan flash full wavelength multifunctional microplate reader (Thermo, USA), a tissue homogenizer (Kinematica, Switzerland), and a 6890n gas chromatograph (Agilent, USA) were used.

### 2.2. Methods

#### 2.2.1. Model Establishment and Grouping

Male Wistar rats were purchased (male, SPF grade, weight 180 ± 20 g, Changchun Yisi Experimental Animal Technology Co., Ltd., license No. 20200034165, License No. SCXK [Ji]-2018-0007), and the animals were reared adaptively for 7 days. Ten rats were randomly selected as the blank group (NC), and the rest of the rats were used to establish the FD model according to the method in “*Methodology of Experimental Animal Models of Traditional Chinese Medicine*” for 14 days. The rats were stimulated with tail clamping twice a day for 25 minutes each time; that is, 1/3 of the tail end was clamped with long thread-removal scissors to make them cry and break free, accompanied by fighting with other rats. A feeding schedule of one-day feeding and two-day fasting was adopted. On the fasting day, gavage was performed with gavage of 2 mL/100 g body weight, twice a day, and water intake was normal. After 14 days of modeling, the food intake of rats returned to normal.

All model rats were randomly divided into a model group (DC: normal saline 1 mL/100 g), a domperidone group (PC: domperidone 2.57 mg/kg), and low-, medium-, and high-dose Kvass groups (GL, GM, and GH: 2, 6, and 18 g/kg). The rats in each group were intragastrically administered a dose of 10 mL/kg body weight. The control group and the model group were given the same amount of distilled water, and each drug group was given the corresponding dose of water solution. The intragastric administration was performed at 8:00 a.m. and 6:00 p.m. daily for 21 days. All animal experiments were carried out in accordance with internationally recognized principles of use and care of laboratory animals, by following the animal experiment methods, ensuring the animal ethics in animal experiments, and minimizing the pain of animals in experiments on the basis of improving efficiency. All experiments were approved by the animal experiment ethics committee of the Harbin University of Commerce.

#### 2.2.2. Behavior Observation and Weight and Food Intake Changes of Rats

The behavior of rats was observed every day, including lazy movement, squint, hair color, weight, and defecation frequency; the rats were fed a weighed solid diet. At 8 a.m. on the next day, the remaining amount of diet was measured. The adaptation period, modeling period, expected dry food intake, and weight change of each rat were calculated.

#### 2.2.3. Detection of Gastric Emptying and Intestinal Propulsion Ratio

After 20 days of administration, all the rats were fasted for 24 hours and were given normal administration on the 21st day. After 30 minutes, the rats in each group were given 5% ink, 3 mL by gavage. After 20 minutes, the rats were killed by cervical spondylectomy; the abdomen was cut open. The stomach was cut along the great curvature, the contents were washed away, and the net weight of the stomach was weighed. The residual rate of gastric contents was calculated according to formula (1).

The small intestine of the rats was taken out and spread on a glass plate without traction. The distance from the pylorus to the ileocecal part was measured as the total length of the small intestine, and the distance from the pylorus to the front of the carbon powder suspension was taken as the propulsion distance of the carbon powder. The propulsion rate of the small intestine was calculated according to equation (2).

(1) $$\begin{array}{c} \text{Gastric residual rate }\left(\%\right)=\frac{A-B}{C+D}\times 100\%, \end{array}$$

where *A* is the total weight of the stomach, *B* is the net weight of the stomach, *C* is the weight of the ink, and *D* is the weight of the drug given

(2) $$\begin{array}{c} \text{Intestinal propulsive rate }\left(\%\right)=\frac{\text{Ink advance distance }\left(\text{cm}\right)}{\text{Total length of small intestine }\left(\text{cm}\right)}\times 100\%. \end{array}$$

#### 2.2.4. Determination of Digestive Enzymes in Rats

The rats in each group were fasted for 24 hours. Then, the rats were anesthetized with ether, the abdominal cavity was cut open, the pylorus was ligated, and the abdominal cavity was sutured quickly. After 3 hours, the rats were killed, the abdominal cavity was cut open. One milliliter of gastric juice was taken and put into a 50 mL conical flask, and then 0.05 mol/L hydrochloric acid solution was added to it and shaken well. The mixed solution was put into two fresh protein tubes, and the bottles were plugged tightly and incubated at 37°C in an incubator for 24 h. Then the protein tubes were taken out, and the length (mm) of the transparent part at both ends of the protein tubes was measured with a Vernier caliper. Pepsin activity and pepsin excretion were calculated.

(3) $$\begin{array}{c} \text{Pepsin activity }\left(\text{U}/\text{mL}\right)={\left(\text{the average length of the transparent part of the four terminal tubules}\right)}^{2}\times 16.\\ \text{Pepsin discharge }\left(\text{U}/\text{h}\right)=\text{pepsin activity}\times \text{gastric juice volume per hour}. \end{array}$$

#### 2.2.5. Determination of Ghrelin, MTL, GAS, and VIP

*(1) Plasma Sample Processing*. After 21 days of intragastric administration, the blood from the posterior ophthalmic venous plexus was taken and bathed in water for 30 min. The levels of ghrelin, MTL, GAS, and VIP in serum samples were detected using an ELISA kit.

*(2) Preparation of Antral Tissue Samples*. After weighing the gastric net weight as mentioned in Section 2.2.4, the antral tissue was quickly cut to about 1 cm in length, washed with 0.9% normal saline, weighed, boiled in 1 mL normal saline at 100°C for 3 min, and then homogenized with 0.5 mL hydrochloric acid (0.1 mol/L). After 1 h at 4°C, 0.5 mL of 0.1 mol/L NaOH was used for neutralization. The supernatant was centrifuged for 30 min at 3000 rpm. The contents of ghrelin, MTL, GAS, and VIP in each tissue sample were detected using an ELISA kit.

#### 2.2.6. Determination of Colon Short-Chain Fatty Acids

According to the method of Yang e al. [27], the contents of the colon were accurately weighed and homogenized with phosphate buffer, centrifuged at 14000 rpm at 4°C for 20 min. Take the supernatant for 0.22 *μ*m water filtration membrane. 400 *μ*L supernatant was extracted with ether for gas phase separation and determination.. The starting temperature of the column was 100°C, which was heated to 140°C at a heating rate of 7.5°C/min and then heated to 200°C at 15°C/min for 3 minutes.

#### 2.2.7. Statistical Analysis

SPSS software was used for statistics. The measurement data were expressed by $\bar{x}\pm s$. A *t*-test was used between the two groups, and the analysis of variance was used between multiple groups. The difference was statistically significant (*P* < 0.05).

## 3. Results

### 3.1. Body Weight and Feed Intake of Rats

As shown in Figure 1, there was no significant difference in weight among all rats during the adaptation period. The body weight of the rats after model building was significantly lower than that of the normal group (*P* < 0.05). After the administration, the weight of rats increased significantly (*P* < 0.05).

As shown in Figure 1, there was no significant difference in food intake among different groups during the adaptation period. After modeling, compared with the blank group, the food intake was significantly reduced (*P* < 0.05). After the intervention, the food intake was significantly higher than that of the model group (*P* < 0.05) and significantly lower than that in the blank group (*P* < 0.05). The intragastric dose level significantly affected the food intake, which was significantly higher in the high-dose group than that in the low-dose group (*P* < 0.05).

### 3.2. Detection of Gastric Residual Rate and Intestinal Propulsion Rate in Rats

The results showed that compared with that of the normal control group, the gastric residual rate of the model group was significantly increased (*P* < 0.05), and compared with that of the model group, the gastric residual rates of the high-, medium-, and low-dose groups were significantly decreased (*P* < 0.05). Compared with that of the normal control group, the intestinal propulsive ratio of the model group was significantly lower (*P* < 0.01), the intestinal propulsive ratios of the medium- and low-dose Kvass groups were significantly lower (*P* < 0.05), and the intestinal propulsive ratios of the positive group and the high-, medium-, and low-dose Kvass groups were significantly higher than that of the model group (*P* < 0.05).

### 3.3. Determination of Digestive Enzymes in Rats

Compared with those in the normal control group, the volumes of gastric juice, pepsin activity, and pepsin excretion in 1 hour in the model group were significantly decreased (*P* < 0.05), and compared with that in the model group, the pepsin excretion in the positive group and the high-dose Kvass group was significantly increased (*P* < 0.05) (Table 1).

### 3.4. Detection of Ghrelin, MTL, GAS, and VIP in Rat Plasma

Compared with those of the normal group, the plasma ghrelin, MTL, and GAS contents of the model group were significantly reduced (*P* < 0.05). Compared with those in the model group, the levels of ghrelin and MTL in the plasma of rats in the Kvass dose group were increased significantly (*P* < 0.05), and the plasma GAS content was increased, but there was no significant difference. The VIP contents of the high-dose group and the medium-dose group were decreased significantly (*P* < 0.05).

### 3.5. Detection of the Contents of Ghrelin, MTL, GAS, and VIP in the Rat Gastric Antrum

The results in Figure 2 show that compared with those of the normal group, the contents of MTL and GAS in the gastric antrum of the model group were significantly decreased (*P* < 0.05), but the content of VIP showed no significant change. Compared with that in the model group, the content of ghrelin in the positive group and the high-dose group was significantly increased (*P* < 0.05), the content of GAS in the high-dose group was significantly increased, and the content of VIP in the medium- and low-dose groups showed no significant change.

### 3.6. Determination of Colon Short-Chain Fatty Acids

As shown in Table 2, the level of total short-chain fatty acids in the colon of the model group was significantly lower than that of the blank group (*P* < 0.05). Compared with those in the model group, except for valeric acid and isovaleric acid, the levels of SCFA and total SCFA in the positive group were significantly increased (*P* < 0.05). The levels of butyric acid and valeric acid in the medium-dose group were higher than those in the low- and high-dose groups. After the intervention, the levels of propionic acid, butyric acid, isobutyric acid, and total SCFA in the high-dose group returned to normal. The results showed that kvass could alleviate the symptoms of FD by regulating the level of short-chain fatty acids in the colon.

## 4. Discussion

Gastrointestinal motility deficiency is an important pathogenesis of FD [17]. The FD rat model was established by starvation and tail clip provocation [6]. It was found that the rat model established by this method had the symptoms of weight loss, delayed gastric emptying, and decreased gastric motility in vitro. After gavage with different doses of kvass, the weight of FD rats increased (Figure 1), gastric emptying rate increased (Figure 3), and gastric motility in vitro increased. The results of this study are basically consistent with those of basic research. Ghrelin is an endogenous ligand that can stimulate food intake and promote gastrointestinal motility [17]. Clinical studies have found that the plasma ghrelin level of FD patients decreased [28]. The results of animal experiments (Figure 2) showed that the content of ghrelin in the plasma of FD model rats decreased significantly, and the content of ghrelin increased after treatment. Studies have shown that FD is associated with decreased MTL release [29, 30]. Compared with the blank group, the content of MTL in the plasma increased significantly, and the content of VIP in the gastric antrum increased significantly, which was similar to the results of Jing et al. [31]. After treatment with kvass, pepsin excretion of rats increased significantly (Table 1). The high-, medium-, and low-dose Kvass groups showed increased levels of SCFA in the colon in varying degrees (Table 2). GAS level may be the pathophysiological mechanism of delayed gastric emptying. In addition, it is reported that the content of GAS in patients with gastric motility disorder may be related to multiple pathogenesis [32, 33]. Reilly et al. [34] reported that short-chain fatty acids instilled into the colon of rats promoted the secretion of GAS in the intestine.

The results showed that kvass could improve the levels of ghrelin, MTL, GAS, and VIP in the serum and gastric antrum, which may be some of the mechanisms of kvass for promoting gastrointestinal motility and treating FD. Kvass can significantly improve the gastrointestinal motility of rats with FD, which lays a preclinical experimental foundation for the use of kvass to alleviate the symptoms of FD. As for the exact mechanism, further experimental research is needed.

## 5. Conclusions

In conclusion, kvass can effectively alleviate the symptoms of food consumption loss and weight loss caused by FD and improve gastrointestinal motility. The increase in pepsin excretion was related to the changes of gastrointestinal hormones and the formation of short-chain fatty acids in the serum and antrum in the presence of gastrointestinal motility disorder. In addition, the beverage can be used as a natural product to alleviate FD.

## Figures and Tables

**Figure 1:** Results of body weight and feed intake in rats ((a) feed intake; (b) body weight). ^∗^Compared with the normal group, the difference was significant (*P* < 0.05). ^∗∗^Significantly different from that of the normal group (*P* < 0.01). ^#^Compared with the model group, the difference was significant (*P* < 0.05).

**Figure 2:** Effect of Kvass on the contents of ghrelin, MTL, GAS, and VIP in rats ((a) effects of Kvass on the contents of ghrelin, MTL, GAS, and VIP in the rat plasma; (b) effects of Kvass on the contents of ghrelin, MTL, GAS, and VIP in the rat gastric antrum).

**Figure 3:** Detection of gastric residual rate and intestinal propulsion rate in rats.

**Table 1:** Determination of digestive enzymes in rats.

Group	Gastric juice volume in 1 h (mL)	Pepsin activity (U/mL)	Pepsin excretion (U/h)
NC	0.83 ± 0.42	463.8 ± 237.0	384.954 ± 99.54
DC	0.55 ± 0.38^∗^	337.4 ± 211.9^∗^	185.57 ± 80.52^∗^
PC	0.79 ± 0.40^#^	433.2 ± 231.4	342.228 ± 92.56^#^
GH	0.77 ± 0.43	404.3 ± 245.5	311.311 ± 105.57^#^
GM	0.68 ± 0.52	399.2 ± 215.6	271.456 ± 112.11^∗^
GL	0.59 ± 0.49	351.9 ± 226.7	207.621 ± 111.08^∗∗^

**Table 2:** Determination of short-chain fatty acids in the colon.

Group	Acetic acid	Propionic acid	Isobutyric acid	Butyrate	Isovaleric acid	Valeric acid	Total SCFA
NC	246.4 ± 42.3	123.8 ± 19.1	27.3 ± 3.1	69.7 ± 16.9	26.9 ± 4.8	23.4 ± 3.7	517.5 ± 89.9
DC	118.3 ± 31.4^∗^	78.9 ± 11.4^∗^	13.4 ± 2.5^∗^	44.1 ± 10.2^∗^	18.3 ± 3.1^∗^	13.3 ± 3.8^∗^	286.3 ± 62.4^∗^
PC	215.1 ± 11.0^#^	141.3 ± 12.9^#^	24.4 ± 2.2^#^	70.4 ± 14.2^#^	19.2 ± 2.9^∗^	17.4 ± 2.9	346.5 ± 33.2^#^
GH	168.4 ± 13.4^∗#^	119.1 ± 13.4	23.7 ± 1.4	63.6 ± 6.9^#^	18.5 ± 1.8^∗^	14.7 ± 1.0^∗^	408 ± 37.9^∗#^
GM	155.7 ± 21.5^∗#^	115.4 ± 19.2^∗#^	22.8 ± 2.1	70.3 ± 11.3^#^	18.7 ± 2.1^∗^	16.3 ± 1.7^∗^	399.2 ± 57.9^∗#^
GL	151.3 ± 22.1^∗#^	113.7 ± 17.3^∗#^	22.9 ± 1.9^∗^	67.0 ± 9.0^#^	20.4 ± 2.8^∗^	15.9 ± 2.4^∗^	391.2 ± 55.5^∗#^

## Data Availability

The datasets generated during and/or analysed during the current study are available from the corresponding authors on reasonable request.
